The article "A Two-Workshop Collaborative, Integrated Scheduling Algorithm considering the Prescheduling of the Root-Subtree Processes" was published in 2022. Journal: Comput Intell Neurosci.

# A Two-Workshop Collaborative, Integrated Scheduling Algorithm considering the Prescheduling of the Root-Subtree Processes

**DOI:** 10.1155/2022/9065638

**Published:** 2022-07-31

**Authors:** Zhiqiang Xie, Haikun Teng, Jingwei Ming, Xiaoguang Yue

**Affiliations:** ^1^College of Computer Science and Technology, Harbin University of Science and Technology, Harbin 150080, China; ^2^Department of Computer Science and Engineering, European University Cyprus, Nicosia 1516, Cyprus

## Abstract

Aiming at the existing two-workshop integrated scheduling algorithm with the same equipment resources, a unified vertical or horizontal scheduling rule is used to sort all processes and ignore the vertical and horizontal characteristics of the associated process position in the process tree, which affects the scheduling results. A two-workshop collaborative, integrated scheduling algorithm considering the prescheduling of the Root-Subtree processes is proposed. The algorithm proposes a process conflict adjustment strategy for the horizontal equipment constraints. The same equipment Root-Subtree processes are sorted and loaded into the corresponding equipment queue through the vertical and horizontal prescheduling method in a single-workshop environment, and it combines with the schedulable process set to dequeue the first process of the queue. To enhance the flexibility of process scheduling, it proposes a process conflict adjustment strategy for the vertical process tree constraints in the two workshops to determine the processing workshop of the processes and the actual start time, which narrows the search comparison for schedulable processes. The example tests show that the algorithm not only excavates and utilizes the effectiveness of the vertical and horizontal characteristics of the process tree, but also considers the process migration time. Therefore, the effect is better and more practical.

## 1. Introduction

The production scheduling problem is to reasonably schedule all data-based processing objects according to production goals and constraints. It is the core content of the current manufacturing research field and belongs to a typical NP-Hard problem. Because the actual industrial production is limited by product structure and manufacturing resources, effective production scheduling can reasonably allocate manufacturing resources and improve the utilization rate of processing equipment. At present, the research on this issue has mainly focused on flow-shop scheduling [1–3] for pure machining or assembly activities without sequence constraints and job-shop scheduling [4–6], as well as integrated scheduling that considers both machining and assembly [7]. Under the current situation of focusing on production efficiency and diversified customization, the manufacturing method of modular design is increasingly favored by more manufacturing enterprises [8–10]. The modularly designed products are composed of multiple modules with closely related parts or components, and the tasks are decomposed from top to bottom. The processing and assembly process with the tree structure constraints is completed. The schematic diagram of the modular product structure is shown in Figure 1. The traditional workshop scheduling method deals with processing and assembly activities separately, which separates the parallel relationship of each processing stage. The integrated scheduling is very prominent in the production of a small or complex product with a tree structure, which is more in line with the actual production needs of manufacturing enterprises. Due to the limitation of various factors such as the large number of parts involved in a single complex product, the different processing attributes, and delivery dates, the collaborative production of two or multiple workshops is considered, which can prevent equipment failure, processing time delays, and other abnormalities. This effectively utilizes idle resources and reduces production costs. At present, the integrated scheduling in single-workshop production has been deeply studied in the general, integrated scheduling, the special constraint relationship, and the flexible equipment [11–15], which is gradually developing in the direction of two workshops or multiworkshops distributed manufacturing [16] according to the actual production demand. As the production fields involved in the integrated scheduling become increasingly extensive, the distributed integrated scheduling for two-workshop collaborative production in the same or different enterprises with the same processing equipment resources has become the research focus. The existing two-workshop integrated scheduling algorithm utilizes the quasi-critical path [17], dynamic critical path [18], and timing strategy [19] to complete all process sequencing and optimize the load balancing [20] and migration times to confirm the process workshop in order to complete the entire product scheduling scheme. However, these algorithms use unified scheduling rules to sort the processing order, making the process scheduling not compact enough and having poor adaptability to process trees of different structures. Additionally, load balance will generate unnecessary idle time periods and limit the number of process migrations, which might reduce the parallel processing capability of processes, making poor results for product scheduling.

Aiming at the above problems, a two-workshop collaborative, integrated scheduling algorithm considering the prescheduling of the Root-Subtree processes (ISA-CPRP) is proposed. Firstly, the preprocessing operation of the simplified decomposition is carried out for the complex product process tree, and the product process tree is divided into several Root-Subtrees using the decomposition granularity control principle. Then, taking the single-workshop production scheduling as the background, the algorithm with the best vertical scheduling effect is used to traverse all Root-Subtrees to obtain the vertical prescheduling completion time, and the algorithm with the best horizontal scheduling effect is used to traverse all the Root-Subtrees to obtain the horizontal prescheduling completion time. According to these prescheduling results, it analyzes the vertical and horizontal characteristics of each Root-Subtree, selects a prescheduling scheme according to the vertical and horizontal characteristics of the Root-Subtree, and determines the priority of each Root-Subtree. Combined with the prescheduling start processing time, all Root-Subtree processes are grouped and sorted in units of the single-workshop processing equipment sequences so that each process can play its own characteristics and end the processing as soon as possible. Finally, the process conflict adjustment strategy of the two-workshop vertical process tree constraints is proposed to determine the process workshop of the process and its actual start time, which discards the equipment balancing strategy, improves the substantial parallel processing capability of the process, and generates a reasonable scheduling scheme for the product in the two workshops with the same equipment resources. The main contributions of this paper are as follows:

- We propose the process conflict adjustment strategy of the horizontal equipment constraints, which excavates the urgency of the product process by the vertical and horizontal prescheduling and achieves both vertical and horizontal process scheduling;
- We propose the process conflict adjustment strategy of the two-workshop vertical process tree constraints, which determines the workshop of the process and start time considering the process migration time and improves the substantial parallel processing capability of the process. This strategy reduces the search and comparison scope of the schedulable process and improves the algorithm solution efficiency and reasonable migration process under the premise of ensuring the completion time.
- The example verification shows that the proposed algorithm can effectively improve the equipment utilization rate and shorten the product processing time in the two-workshop integrated scheduling, and it can be well applied to the product examples of different structures.

## 2. Related Works

This section reviews the related works about the two-workshop integrated scheduling algorithm to solve the problem of the two-workshop integrated scheduling. The methods can divide into three categories: the vertical or horizontal optimization strategy-based methods, the workshop balance strategy-based methods, and the meta-heuristic algorithm-based methods. The horizontal optimization strategy-based methods such as ISA-EPSP [21] adopt the schedulable process workshop balance strategy for grouping and determine the processing workshop of the process according to the grouped process workshop strategy, which is a horizontal overall optimization method. The algorithm (ISA-TWOT) in [22] adopts the idea of time-selected two-workshop scheduling and proposes a process sequence sorting strategy, which starts from the overall structure of the process tree and forms an initial scheduling scheme by selecting a long path. The algorithm (ISA-TPNR) in [23] proposes a key equipment balancing strategy, a neighborhood rendering strategy, and a process workshop selection strategy with the same equipment, which are used to determine the processing workshop for the processes. It uses the dynamic critical path strategy and the short time strategy to determine the process scheduling sequence and the start processing time. The meta-heuristic algorithm-based methods such as ISA-AEMA [24] adopt a meta-heuristic algorithm to solve the multiworkshop collaborative, integrated scheduling problem, which is analyzed on the whole under the premise of satisfying the constraints, and a feasible solution is obtained through multiple iterations. From the above analysis, the existing rule-based two-workshop integrated scheduling algorithms use unified scheduling rules to analyze and sort all processes in the product process tree. Each scheduling requires numerous searches and comparisons of all schedulable processes to determine the final processing workshop and actual processing time of the process. The vertical and horizontal characteristics of the process in the partial order relationship in the product process tree are ignored so that the processing process of the product is not compact enough, and the scheduling result is greatly restricted by the product structure. At the same time, the load balancing and migration times between the two workshops are considered the main optimization goals, but the real goal of the coordinated, integrated scheduling of the two workshops is to shorten the product processing time, not to evenly distribute the processing tasks to two workshops with the same equipment resources; the load balancing processing strategy will increase the number of unnecessary migrations and affect the scheduling result. Because the total time for manufacturing products is limited by the vertical and horizontal aspects of the process tree and processing equipment, at the same time, the different product structures lead to different vertical and horizontal characteristics of the process tree's internal partial order relationship. Therefore, it is necessary to study the integrated scheduling problem of the vertical and horizontal characteristics inside the product process tree, which provides a new research direction for solving the distributed integrated scheduling problem of complex products. Currently, there is no research result of the distributed integrated scheduling algorithm for the vertical and horizontal characteristic analysis inside the product process tree.

## 3. Description of the Problem Model

The two-workshop collaborative, integrated scheduling is to study the collaborative production scheduling problem of two workshops with the same equipment resources on the basis of the general, integrated scheduling, so the vertical and horizontal coordination requirements for the algorithm scheduling are higher. The integrated scheduling problem is mainly aimed at the product process diagram with a tree structure, which is consistent with the production task decomposition structure of the distributed modular design, each leaf node represents the information of the process, and the directed edge represents the partial order relationship between the processes. The leaf node is the start point of the product processing scheduling, and the root node is the end point of the product processing scheduling. Because a complex product will cause excessive load on the workshop equipment in the actual production, to make full use of the idle resources and shorten the total processing time of the product to ensure the delivery time, the processes need to be coordinated and scheduled between the two workshops. The transfer time of the process between two workshops is called the operation migration time. The processing or assembling processes are collectively referred to as the processing processes, and the related equipment is collectively referred to as the processing equipment. The two-workshop collaborative, integrated scheduling not only has the generality of the general single-workshop integrated scheduling, but also has its own particularity, which is mainly reflected in that when two processes with partial order relationship are not processed in the same workshop, the process migration time needs to be considered. Therefore, the two-workshop collaborative, integrated scheduling problem needs to meet the following constraints: ① only one process can be processed on one processing equipment at the same time period; ② each process can only be continuously processed on one processing equipment in one workshop and cannot be interrupted after being processed; ③ the processing sequence of the process must meet the constraints of the process tree; ④ it allows the processing equipment to be idle, and the process can be processed after the processing equipment is idle; ⑤ if the process and its immediately following processes are not processed in the same workshop, the immediately following process will cause the process migration; and ⑥ the processing time of each process is fixed, and the process migration time is fixed. In order to facilitate the description of the scheduling algorithm in this paper, the relevant definitions are described as follows:

**Definition 1 .**

Root-Subtree set: it takes out the root node and splits the process tree into more than two Root-Subtrees through the decomposition granularity control principle.

**Definition 2 .**

Vertical prescheduling completion time: it schedules the completion processing time of each Root-Subtree through the algorithm ① “dynamic critical path, short time” strategy in the single-workshop environment.

**Definition 3 .**

Horizontal prescheduling completion time: it schedules the completion processing time of each Root-Subtree through the algorithm ② “layer priority, short time, long path” strategy in the single-workshop environment.

**Definition 4 .**

Root-Subtree priority: it uses the vertical and horizontal advantages of the Root-Subtree to analyze the results and sets the parameters of the Root-Subtree scheduling priority through the selected Root-Subtree prescheduling completion time from large to small.

**Definition 5 .**

Process migration time: the time period required for a process to be moved from one workshop to another.

**Definition 6 .**

Prescheduling start processing time: during the analysis of the vertical and horizontal advantages of the Root-Subtree, the start processing time of each Root-Subtree process on the corresponding processing equipment is obtained according to the selected prescheduling scheme.

Assuming that a product consists of *n* processes, its product process tree can be split into *N* Root-Subtrees, and collaborative processing is planned in workshop W1 and workshop W2 with the same equipment resources. Each workshop has a total of m processing equipment. The process migration time between the two workshops is *T*_*pm*_, and the early completion of the product requires each process to start processing as soon as possible. Although there is no direct relationship between the number of migrations and the total processing time of the product, effectively controlling migration can reduce additional production costs. The objective and constraint functions of the problem are as follows:

(1) $$\begin{array}{c} T=\min\left\{\max\left\{S_{i,j}^{a}+T_{i,j}\right\}\right\}, \end{array}$$

(2) $$\begin{array}{c} \text{s.t.}\min\left\{S_{i,j}^{a}\right\}, \end{array}$$

(3) $$\begin{array}{c} F_{i,j}^{w}=S_{i,j}^{a}+T_{i,j}, \end{array}$$

(4) $$\begin{array}{c} S_{x,y}^{a}\geq F_{i,j}^{w}, \end{array}$$

(5) $$\begin{array}{c} S_{i,j}^{a}\geq F_{j}^{w}.\max, \end{array}$$

(6) $$\begin{array}{c} F_{j}^{c}.\max-F_{x,y}^{w}\left\{\begin{array}{c} \geq T_{pm}\\ <T_{pm} \end{array}\right., \end{array}$$

(7) $$\begin{array}{c} \frac{T_{Z}^{rt_{k}}}{T_{H}^{rt_{k}}}\left\{\begin{array}{c} >1\\ =1\\ <1 \end{array}.\right. \end{array}$$

In the above formula, *T* represents the completion time of all the product processes; *S*_*i*,*j*_^*a*^ represents the actual start processing time of process *i* on the processing equipment *j*; *T*_*i*,*j*_ represents the continuous processing time of process *i* on the processing equipment *j*; *w* represents the workshop number, *c* represents another workshop number; *F*_*i*,*j*_^*w*^ represents the completion time of process *i* on processing equipment *j* of workshop *w*; *F*_*j*_^*w*^.max represents the last completion time on the processing equipment *j* of workshop *w* at the current moment; *T*_*Z*_^*rt*_*k*_^ represents the completion time of the Root-Subtree *rt*_*k*_ vertical prescheduling, *T*_*H*_^*rt*_*k*_^ represents the completion time of the Root-Subtree *rt*_*k*_ horizontal prescheduling, and *rt*_*k*_ is the *k* Root-Subtree of the product process tree, 1 ≤ *k* ≤ *N*. Formula (1) is the optimization goal of the proposed algorithm, and the product will be completed as soon as possible. Formula (2) indicates that each process can start processing as early as possible on the workshop equipment. Formula (3) indicates that each process is continuously processed on the workshop equipment and cannot be interrupted once processed. Formula (4) indicates that each process must comply with the scheduling constraints of the process tree. In other words, the actual start processing time of each process should be greater than the processing completion of all its immediately preceding processes. Formula (5) indicates that the actual start processing time of the process must be greater than or equal to the final completion time of all immediately preceding processes with the same equipment. Formula (6) indicates that when the process is migrated, if the difference between the last end time of the processing equipment and the immediately preceding process end time of the currently scheduled process is greater than or equal to the process migration time, then the process migration time is ignored, if it is less than the process migration time, the process migration time will be considered in the process of calculating the actual start processing time of the current schedulable process. Formula (7) represents the ratio of the vertical prescheduling completion time of the Root-Subtree *rt*_*k*_ to the horizontal prescheduling completion time. When the result is less than 1, the Root-Subtree has the advantage of vertical characteristics, and the algorithm ① prescheduling scheme is selected as the reference scheme for the vertical and horizontal characteristics of the Root-Subtree. When the result is greater than 1, the Root-Subtree has the advantage of horizontal characteristics, and the algorithm ② prescheduling scheme is selected as the reference scheme for the vertical and horizontal characteristics of the Root-Subtree. When the result is equal to 1, the Root-Subtree has the vertical and horizontal balance characteristics, and the prescheduling scheme of algorithm ① or algorithm ② can be used as a reference scheme for the vertical and horizontal characteristics of the Root-Subtree. To simplify the algorithm complexity, this study directly determines the Root-Subtree with both vertical and horizontal advantages as the vertical advantage.

## 4. Problem Analysis and Algorithm Strategy Design

### 4.1. Design of the Process Conflict Adjustment Strategy of the Horizontal Equipment Constraints

#### 4.1.1. Design of the Root-Subtree Priority Strategy

In order to mine the vertical and horizontal characteristics of the associated position of the process inside the process tree, this paper needs to preprocess the process tree. The process tree decomposition preprocessing is to split the process tree into several independent subtrees according to certain decomposition subtree granularity rules. If the granularity is too coarse, the vertical and horizontal characteristics of the internal structure of the process tree cannot be obtained. If the granularity is too fine, the decomposition process will be very complicated, which will greatly increase the fusion cost between subtrees, so the decomposition subtree granularity rule is to split the process tree into several Root-Subtrees to form a Root-Subtree set. When the product is modularly designed, the structural characteristics of different products have different process tree models [25]. In other words, in the integrated scheduling product process tree model, there may be a special case where the in-degree of the root node is not greater than 1, so that the process tree cannot be directly split into the Root-Subtree set from the root node. Therefore, when the product process tree is split according to the decomposition granularity control principle, firstly, it is necessary to judge whether the in-degree of the root node is greater than 1 in reverse order. If the in-degree of the root node is 1, it judges whether the in-degree of the immediately preceding process of the root node is greater than 1, with loop judgment until the process with the first occurrence of the in-degree greater than 1 is found. The process and all its direct or indirect immediately following processes are sequentially pushed into the stack according to the judgment order, and the other remaining processes form a Root-Subtree set on the basis of maintaining the original partial order relationship of the process tree. According to the process tree structure, the Root-Subtrees are named from left to right as *rt*_1_, *rt*_2_, *rt*_3_,…, *rt*_*N*_. There is a product process tree O, and its splitting process schematic diagram is shown in Figure 2, where the in-degree of the root node process O1 is 1. The in-degree of its immediately preceding process O2 is 3, so processes O1 and O2 are taken out and placed on the stack according to the judgment order, and all remaining nodes form a Root-Subtree set on the basis of retaining the original constraint relationship. In other words, the four processes O3, O6, O7, and O10 form the Root-Subtree *rt*_1_; the three processes O4, O8, and O11 form the Root-Subtree *rt*_2_; the four processes O5, O9, O12, and O13 form the Root-Subtree *rt*_3_; and the decomposition of the product process tree is completed.

After the Root-Subtree set is formed, in a single-workshop environment, each Root-Subtree is traversed through algorithm ① to obtain the vertical prescheduling completion time, and each Root-Subtree is traversed through algorithm ② to obtain the horizontal prescheduling completion time. Scheduling at this time is not the real production scheduling. It is only used as a reference for analyzing the vertical and horizontal characteristics of the Root-Subtree. It compares the prescheduling completion time of algorithm ① and algorithm ② to determine whether the Root-Subtree has a vertical advantage or a horizontal advantage. Because the Root-Subtree set is a subtree inside the product, it has the same optimization goal as the product itself. By using this criterion, the scheduling scheme with the short prescheduling completion time is selected as the reference scheme for the vertical and horizontal advantages of the Root-Subtree, that is, min{*T*_*Z*_^*rt*_*k*_^, *T*_*H*_^*rt*_*k*_^},  1 ≤ *k* ≤ *N*. Formula (7) is used as the objective function to analyze the vertical and horizontal characteristics of the Root-Subtree. Compared with the quasi-critical path of the product process tree, the Root-Subtree is a branch of the product process tree, and the prescheduling completion time of the Root-Subtree can better indicate the lower limit of the product scheduling completion time. When two or more Root-Subtrees have the same prescheduling completion time, the Root-Subtree with more processes has a higher priority. When the number of the processes is the same,the priority is set according to the naming order of the Root-Subtree. The Root-Subtree priority strategy is ready to solve the problem of scheduling conflicts in the Root-Subtree process on the same equipment [26, 27]. Even if all Root-Subtrees have uniform vertical and horizontal characteristics, the Root-Subtree priority strategy can better illustrate the process scheduling urgency than the quasi-critical path or long path strategy.

The product process tree O of Figure 2 is taken as an example. It specifically analyzes the vertical and horizontal characteristics of the Root-Subtree *rt*_1_ and determines the priority of the three Root-Subtrees. It uses algorithm ① and algorithm ② to preschedule the Root-Subtree *rt*_1_ to get the vertical prescheduling completion time *T*_*Z*_^*rt*_1_^=95 and the horizontal prescheduling completion time *T*_*Z*_^*rt*_1_^=75. The vertical and horizontal comparison of the prescheduling Gantt chart is shown in Figure 3(a). According to the comparison results of *T*_*Z*_^*rt*_1_^/*T*_*H*_^*rt*_1_^ > 1, the Root-Subtree *rt*_1_ has a horizontal advantage, which indicates that the compactness of the Root-Subtree process is better when the horizontal scheduling is the main method, so that the prescheduling completion time *T*_*Z*_^*rt*_1_^=75 is determined as the reference time for setting the priority of the Root-Subtree *rt*_1_. In the same way, the reference times for setting the priority of the Root-Subtrees *rt*_2_ and *rt*_3_ are *T*_*Z*_^*rt*_2_^=*T*_*H*_^*rt*_2_^=60 (the Root-Subtree has vertical and horizontal balance characteristics) and *T*_*Z*_^*rt*_3_^=90 (the Root-Subtree has a vertical advantage), and the vertical and horizontal comparison of the Root-Subtree *rt*_2_ and *rt*_3_ prescheduling Gantt charts are shown in Figures 3(b) and 3(c). The priority of each Root-Subtree is determined through the above analysis, that is, *Q*_*rt*_^1^=*T*_*Z*_^*rt*_3_^=90, *Q*_*rt*_^2^=*T*_*Z*_^*rt*_1_^=75, and *Q*_*rt*_^3^=*T*_*Z*_^*rt*_3_^=60. It shows that the Root-Subtree *rt*_3_ has the highest priority in the scheduling fusion of the Root-Subtree process, and the prescheduling scheme of algorithm ② is the selected reference scheme. The priority of the Root-Subtree *rt*_1_ is the second, and the prescheduling scheme of algorithm ① is the selected reference scheme. Root-Subtree *rt*_2_ has the lowest priority, and the prescheduling scheme of algorithm ① is the selected reference scheme.

#### 4.1.2. Design of the Same Equipment Root-Subtree Process Sorting Strategy

Whether it is the traditional single-workshop integrated scheduling or the distributed two-workshop collaborative, integrated scheduling, the process scheduling will have the competition problem for the processing equipment resources. Therefore, this paper needs to design the same equipment Root-Subtree process sorting strategy based on the analysis of the Root-Subtree vertical and horizontal characteristics. Combined with the priority parameters of the Root-Subtree, the Root-Subtree process scheduling order on the horizontal processing equipment is determined. It makes full use of the vertical and horizontal advantages of each branch inside the process tree to seek a more reasonable scheduling processing sequence for the processes and improves the compactness of the Root-Subtree process scheduling. In the single-workshop environment, the same equipment Root-Subtree process sorting strategy is used to obtain the prescheduling start processing time of each Root-Subtree process with the help of the selected Root-Subtree prescheduling scheme, and the Root-Subtree process sequence of the same equipment is determined by comparing the prescheduling start processing time. In this paper, the single-workshop equipment sequence is used as the Root-Subtree process to establish a grouping, and the scheduling order of all Root-Subtree processes on the corresponding processing equipment is determined according to the prescheduling start processing time from small to large. The Root-Subtree processes in the earlier order are prioritized, and the urgency of the Root-Subtree processes is fully exploited, which is in line with the concept of early processing and early completion of the integrated scheduling. When multiple processes of the same equipment have the same prescheduling start processing time, the high-priority Root-Subtree process has a greater impact on the lower limit of the product scheduling completion time. The process with higher Root-Subtree priority is prioritized in the fusion scheduling process, which makes subsequent processes become schedulable processes earlier and enhances the process scheduling compactness. This situation can only occur between different Root-Subtrees.

By taking the product process tree O in Figure 2 as an example, three groups are established for the Root-Subtree processes on the equipment M1, M2, and M3, and the prescheduling start processing time of each Root-Subtree process is determined according to the prescheduling scheme selected by the vertical and horizontal advantages of the Root-Subtree itself. It specifically analyzes the ordering process of the Root-Subtree processes on the equipment M1. Figures 3(a)–3(c)show that the Root-Subtree processes processed on equipment M1 and its corresponding prescheduling start processing time are {O6:10, O8:20, O9:20, O13:0}, where the prescheduling start processing time of processes O8 and O9 are both 20. Because the priority of the Root-Subtree to which process O8 belongs is lower than the priority of the Root-Subtree to which process O9 belongs, process O9 is scheduled preferentially. Therefore, using the same Root-Subtree process sorting strategy, the Root-Subtree process scheduling sequence of equipment M1 is obtained as O13⟶O6⟶O9⟶O8. In the same way, all Root-Subtree processes of the product process tree O are grouped and sorted in units of the single-workshop processing equipment sequences, as shown in Table 1.

### 4.2. Design of the Process Conflict Adjustment Strategy of the Two-Workshop Vertical Process Tree Constraints

In the process from the independent prescheduling of the Root-Subtree set to the overall substantive scheduling, all Root-Subtree processes need to meet the vertical and horizontal constraints of the integrated scheduling. The process conflict adjustment strategy of the horizontal equipment constraints solves the problem of the horizontal processing equipment competition. Therefore, this section proposes the process conflict adjustment strategy of the two-workshop vertical process tree constraints to solve the scheduling sequence constraint problem of all processes in the vertical process tree. After the same equipment Root-Subtree process scheduling sequence is formed, the two-workshop collaborative, integrated scheduling problem mainly focuses on selecting a suitable processing workshop and determining a reasonable start processing time, which further improves the parallelism and compactness of the process scheduling and avoids falling into the local optimal [28]. Firstly, it sets two workshops: the master workshop and the slave workshop. The product processing task starts with the master workshop to prepare for how to select a processing workshop under the same conditions. The start time of the entire product processing is 0. It establishes a set of queues corresponding to the processing equipment in the single workshop and loads the same equipment Root-Subtree processes into the corresponding queue in order from front to back according to the scheduling order determined by the process conflict adjustment strategy of the horizontal equipment constraints. Due to the particularity of the two-workshop collaborative production, the process can be selected and processed on two processing equipment with the same function. In other words, in each scheduling calculation process, the process has two final completion times that need to be considered. In order to ensure the uniqueness of the process's initial start processing time, this paper uses the mathematical relationship between the processing completion time of the immediately preceding process and the process migration time in the process tree of the current schedulable process as the initial start processing time of the process. It should be emphasized that the initial start processing time of the independent process is 0 by default. Then, considering the process migration time, the two final completion times of the equipment with the same function in the two workshops are compared with the initial start processing time of the first process of the queue. It uses the integrated scheduling concept of early processing and early completion to determine the processing workshop of the process and its actual start processing time and generates the substantial scheduling scheme of the Root-Subtree process in the two-workshop environment. Finally, all non-Root-Subtree processes are popped out of the stack and scheduled to form a final scheduling scheme to complete the product processing task. In order to fully describe the strategy, it supposes that there is schedulable process *p*_*i*,*j*_, the initial start processing time is *S*_*i*,*j*_^*s*^, the actual start processing time is *S*_*i*,*j*_^*a*^, the two final completion times of the two-workshop processing equipment *j* corresponding to process *p*_*i*,*j*_ are, respectively, *F*_*j*_^*W*1^.max and *F*_*j*_^*W*2^.max, the two reference start processing times of the two-workshop processing equipment *j* corresponding to process *p*_*i*,*j*_ are, respectively, *S*_*i*,*j*_^*W*1^ and *S*_*i*,*j*_^*W*2^, and the process migration time of the two workshops is *T*_*pm*_. The following describes how to scientifically and rationally select the processing workshop of the process and determine the actual start processing time of the process under the environment of the two workshops with the same equipment resources (workshop W1 is the main workshop, and workshop W2 is the slave workshop). There are the following situations:

  Situation 1. The schedulable process *p*_*i*,*j*_ is independent. Because the process has no immediately preceding process, there is no need to consider the process migration problem and *S*_*i*,*j*_^*s*^ = 0. There are three forms to consider in this case: 1) if *F*_*j*_^*W*1^.max < *F*_*j*_^*W*2^.max, process *p*_*i*,*j*_ is assigned to workshop W1 and *S*_*i*,*j*_^*a*^ = *F*_*j*_^*W*1^.max; 2) if *F*_*j*_^*W*1^.max > *F*_*j*_^*W*2^.max, process *p*_*i*,*j*_ is assigned to workshop W2 and *S*_*i*,*j*_^*a*^ = *F*_*j*_^*W*2^.max; and3) if *F*_*j*_^*W*1^.max = *F*_*j*_^*W*2^.max, process *p*_*i*,*j*_ is assigned to the master workshop W1 and *S*_*i*,*j*_^*a*^ = *F*_*j*_^*W*1^.max, so that more idle time can be reserved for the slave workshop W2.
  Situation 2. The schedulable process *p*_*i*,*j*_ has an immediately preceding process, and the relationship between the initial start processing time and the two final completion times of the corresponding two-workshop processing equipment is *S*_*i*,*j*_^*s*^ ≤ min{*F*_*j*_^*W*1^.max, *F*_*j*_^*W*2^.max}. (1) When *F*_*j*_^*W*1^.max = *F*_*j*_^*W*2^.max, this situation needs to consider two forms: ① when *F*_*j*_^*W*1^.max − *S*_*i*,*j*_^*s*^ ≥ *T*_*pm*_, process *p*_*i*,*j*_ is assigned to workshop W1 and *S*_*i*,*j*_^*a*^ = *F*_*j*_^*W*1^.max; ② when *F*_*j*_^*W*1^.max − *S*_*i*,*j*_^*s*^ < *T*_*pm*_, if the immediately preceding process of the process *p*_*i*,*j*_ is processed in workshop W1, process *p*_*i*,*j*_ is assigned to workshop W1 and *S*_*i*,*j*_^*a*^ = *F*_*j*_^*W*1^.max, and if the immediately preceding process of the process *p*_*i*,*j*_ is processed in workshop W2, process *p*_*i*,*j*_ is assigned to workshop W2 and *S*_*i*,*j*_^*a*^ = *F*_*j*_^*W*2^.max. (2) When *F*_*j*_^*W*1^.max < *F*_*j*_^*W*2^.max, this situation needs to consider two forms: ① if the immediately preceding process of the process *p*_*i*,*j*_ is processed in the workshop W1, process *p*_*i*,*j*_ is assigned to workshop W1 and *S*_*i*,*j*_^*a*^ = *F*_*j*_^*W*1^.max; ② it assumes that the immediately preceding process of process *p*_*i*,*j*_ is processed in workshop W2. If process *p*_*i*,*j*_ is assigned to workshop W2, the process migration does not need to be considered, and the reference start processing time in workshop W2 is *S*_*i*,*j*_^*W*2^ = *F*_*j*_^*W*2^.max. If process *p*_*i*,*j*_ is assigned to workshop W1, and the process migration problem needs to be considered at this time, it is necessary to calculate the difference between *F*_*j*_^*W*1^.max in workshop W1 and the initial start processing time *S*_*i*,*j*_^*s*^ of process *p*_*i*,*j*_, when *F*_*j*_^*W*1^.max − *S*_*i*,*j*_^*s*^ ≥ *T*_*pm*_. It is not necessary to consider the process migration, and the reference start processing time of process *p*_*i*,*j*_ in workshop W1 is *S*_*i*,*j*_^*W*1^ = *F*_*j*_^*W*1^.max. At this time *S*_*i*,*j*_^*W*1^ < *S*_*i*,*j*_^*W*2^; therefore, process *p*_*i*,*j*_ is finally assigned to workshop W1 and *S*_*i*,*j*_^*a*^ = *S*_*i*,*j*_^*W*1^. When *F*_*j*_^*W*1^.max − *S*_*i*,*j*_^*s*^ < *T*_*pm*_, the process migration needs to be considered, the reference start processing time of the process *p*_*i*,*j*_ in workshop W1 is *S*_*i*,*j*_^*W*1^ = *F*_*j*_^*W*1^.max + *T*_*pm*_ − (*F*_*j*_^*W*1^.max − *S*_*i*,*j*_^*s*^). Then, the reference start processing time of process *p*_*i*,*j*_ in the two workshops are compared. If *S*_*i*,*j*_^*W*1^ < *S*_*i*,*j*_^*W*2^, process *p*_*i*,*j*_ is finally assigned to workshop W1 and *S*_*i*,*j*_^*a*^ = *S*_*i*,*j*_^*W*1^. Otherwise, process *p*_*i*,*j*_ is finally assigned to workshop W2 and *S*_*i*,*j*_^*a*^ = *S*_*i*,*j*_^*W*2^. Similarly, when *F*_*j*_^*W*1^.max > *F*_*j*_^*W*2^.max, the analysis process is the same as described above.
  Situation 3. The schedulable process *p*_*i*,*j*_ has an immediately preceding process, and the relationship between the initial start processing time and the two final completion times of the corresponding two-workshop processing equipment is *F*_*j*_^*W*1^.*max* < *S*_*i*,*j*_^*s*^ < *F*_*j*_^*W*2^.*max*. There are two forms to consider in this case: ① when the immediately preceding process of process *p*_*i*,*j*_ is processed in workshop W1, process *p*_*i*,*j*_ is assigned to workshop W1, and *S*_*i*,*j*_^*a*^ = *S*_*i*,*j*_^*s*^, there is no need to consider the process migration, and the actual start processing time of the process is the earliest and ② when the immediately preceding process of process *p*_*i*,*j*_ is processed in the workshop W2, it is necessary to judge whether the reference processing start time *S*_*i*,*j*_^*W*1^ = *S*_*i*,*j*_^*s*^ + *T*_*pm*_ of process *p*_*i*,*j*_ in workshop W1 is less than the reference processing start time *S*_*i*,*j*_^*W*2^ = *F*_*j*_^*W*2^.*max* in workshop W2. If *S*_*i*,*j*_^*W*1^ < *S*_*i*,*j*_^*W*2^, process *p*_*i*,*j*_ is assigned to workshop W1 and *S*_*i*,*j*_^*a*^ = *S*_*i*,*j*_^*W*1^. Otherwise, process *p*_*i*,*j*_ is assigned to workshop W2 and *S*_*i*,*j*_^*a*^ = *S*_*i*,*j*_^*W*2^. Similarly, when the relationship between the initial start processing time of process *p*_*i*,*j*_ and the two final completion times of the corresponding two-workshop processing equipment is *F*_*j*_^*W*2^.*max* < *S*_*i*,*j*_^*s*^ < *F*_*j*_^*W*1^.*max*, the analysis process is the same as the above description.
  Situation 4. The schedulable process *p*_*i*,*j*_ has an immediately preceding process, and the relationship between the initial start processing time and the two final completion times of the corresponding two-workshop processing equipment is *S*_*i*,*j*_^*s*^ ≥ *max*{*F*_*j*_^*W*1^.*max*, *F*_*j*_^*W*2^.*max*}. If the immediately preceding process of process *p*_*i*,*j*_ is processed in workshop W1, the reference start processing time in workshop W1 is *S*_*i*,*j*_^*W*1^ = *S*_*i*,*j*_^*s*^, and the reference processing start time of process *p*_*i*,*j*_ in workshop W2 is *S*_*i*,*j*_^*W*2^ = *S*_*i*,*j*_^*s*^ + *T*_*pm*_. Because *S*_*i*,*j*_^*W*1^ < *S*_*i*,*j*_^*W*2^, the process *p*_*i*,*j*_ is finally assigned to workshop W1 and *S*_*i*,*j*_^*a*^ = *S*_*i*,*j*_^*s*^. Similarly, if the immediately preceding process of process *p*_*i*,*j*_ is processed in workshop W2, the analysis process is the same as that described above.
  Situation 5. The schedulable process *p*_*i*,*j*_ has two immediately preceding processes {*p*_*x*,*y*_, *p*_*u*,*v*_} in the process tree: (1) when two immediately preceding processes are processed in the same workshop, the initial start processing time of the process *p*_*i*,*j*_ is *S*_*i*,*j*_^*s*^ = max{*F*_*x*,*y*_^*w*^, *F*_*u*,*v*_^*w*^} and (2) when the two immediately preceding processes are not processed in the same workshop, the initial start processing time of process *p*_*i*,*j*_ needs to be obtained according to the actual form. It assumes that the processing completion time *F*_*x*,*y*_^*W*1^ of process *p*_*x*,*y*_ in workshop W1 is less than the processing completion time *F*_*u*,*v*_^*W*2^ of process *p*_*u*,*v*_ in workshop W2. There are two forms to consider in this case: ① if *F*_*u*,*v*_^*W*2^ − *F*_*x*,*y*_^*W*1^ is greater than or equal to the process migration time *T*_*pm*_, the initial start processing time of process *p*_*i*,*j*_ is *S*_*i*,*j*_^*s*^ = *F*_*u*,*v*_^*W*2^ and ② if *F*_*u*,*v*_^*W*2^ − *F*_*x*,*y*_^*W*1^ is less than the process transition time *T*_*pm*_, the initial start processing time of process *p*_*i*,*j*_ is *S*_*i*,*j*_^*s*^ = *F*_*u*,*v*_^*W*2^ + *T*_*pm*_ − (*F*_*u*,*v*_^*W*2^ − *F*_*x*,*y*_^*W*1^). Similarly, when the processing completion time *F*_*x*,*y*_^*W*1^ of process *p*_*x*,*y*_ in workshop W1 is greater than the processing completion time *F*_*u*,*v*_^*W*2^ of process *p*_*u*,*v*_ in workshop W2, the analysis process is the same as the above description. After the initial start processing time of process *p*_*i*,*j*_ is determined, how to select the processing workshop of the process and determine the actual start processing time of the process is analyzed according to situation 2, situation 3, or situation 4. The above analysis method can be extended to the situation where two or more immediately preceding processes are processed in the same or different workshops.

The algorithm flowchart of the process conflict adjustment strategy of the two-workshop vertical process tree constraints is shown in Figure 4. The specific implementation steps are as follows:

  Step 1: it determines whether the first process of queues **Q** is a schedulable process according to the schedulable process set. If no, the first process of the queue does not perform the dequeue operation. If yes, go to step 2.
  Step 2: it determines whether the first process of the queue is independent. If yes, the initial start processing time of the first process of the queue is *S*_*i*,*j*_^*s*^=0. According to the analysis process of situation 1, it determines the processing workshop of the process and its actual start processing time, and the first process of the queue is dequeued and scheduled; go to step 8. If no, go to step 3.
  Step 3: it determines whether the number of the immediately preceding process of the first process of the queue is 1. If yes, the initial start processing time *S*_*i*,*j*_^*s*^ of the first process of the queue is the processing completion time of the immediately preceding process; go to step 4. If no, go to step 7.
  Step 4: it determines whether the initial start processing time *S*_*i*,*j*_^*s*^ of the first process of the queue is less than min{*F*_*j*_^*W*1^.max, *F*_*j*_^*W*2^.max}. If yes, it determines the processing workshop of the process and its actual start processing time according to the analysis process of situation 2, and the first process of the queue is dequeued and scheduled; go to step 8. If no, go to step 5.
  Step 5: it determines whether the starting processing time *S*_*i*,*j*_^*s*^ of the first process of the queue is greater than *F*_*j*_^*W*1^.max and less than *F*_*j*_^*W*2^.max. If yes, it determines the processing workshop of the process and its actual starting processing time according to the analysis process of situation 3, and the first process of the queue is dequeued and scheduled, go to step 8. If no, go to step 6.
  Step 6: the initial start processing time *S*_*i*,*j*_^*s*^ of the first process of the queue is greater than or equal to max{*F*_*j*_^*W*1^.max, *F*_*j*_^*W*2^.max}. According to the analysis process of situation 4, the processing workshop of the process and its actual start processing time are determined, and the first process of the queue is dequeued and scheduled; go to step 8.
  Step 7: the number of the immediately preceding process of the first process of the queue is greater than 1. It determines the initial start processing time *S*_*i*,*j*_^*s*^ of the first process of the queue according to situation 5; go to step 4.
  Step 8: it deletes the scheduled processes from the schedulable process set and adds the new schedulable process to the schedulable process set **P**.

## 5. Algorithm Detailed Design and Complexity Analysis

### 5.1. Algorithm Detailed Design

The algorithm flowchart of a two-workshop collaborative, integrated scheduling algorithm considering the prescheduling of the Root-Subtree processes is shown in Figure 5. The specific implementation steps are as follows:

  Step 1: it processes data information for the processing and assembling process of the complex products and forms a standardized integrated scheduling process tree model.
  Step 2: it determines whether the in-degree of the root node of the product process tree is greater than 1. If no, go to step 3. If yes, take out the root node, store it in the stack space, and go to step 4.
  Step 3: the root node is taken out and stored in the stack space, and the immediately preceding process of the original root node becomes the new root node of the process tree. It determines whether the root node has an immediately preceding process. If yes, go to step 2. If no, go to step 15.
  Step 4: according to the decomposition granularity control principle, the product process tree is divided into several Root-Subtrees to form a Root-Subtree set {*rt*_1_, *rt*_2_, *rt*_3_,…, *rt*_*N*_}.
  Step 5: the vertical prescheduling completion time *T*_*Z*_^*rt*_*k*_^ and the horizontal prescheduling completion time *T*_*H*_^*rt*_*k*_^ of each Root-Subtree are obtained by the prescheduling method.
  Step 6: according to whether the comparison result of step 5 is less than or equal to 1, it determines the vertical and horizontal advantages of the Root-Subtree. If yes, the vertical scheduling scheme is selected. If no, the horizontal prescheduling scheme is selected.
  Step 7: according to the selected prescheduling scheme in step 6, the prescheduling completion time corresponding to the Root-Subtree and the prescheduling start processing time of all Root-Subtree processes are obtained.
  Step 8: it uses the prescheduling completion time selected by the Root-Subtree and the bubble sort to determine each Root-Subtree priority parameter. All the Root-Subtrees are marked from high to low.
  Step 9: all the Root-Subtree processes are grouped according to the single-workshop equipment sequence, and it sorts the Root-Subtree processes according to the prescheduled start processing time and the Root-Subtree priority parameters.
  Step 10: it establishes a set of queues **Q** corresponding to the single-workshop equipment sequence and loads the same equipment Root-Subtree processes into the corresponding queues from front to back according to the scheduling order determined in step 9.
  Step 11: it establishes a schedulable process set **P** and adds all schedulable processes in the product process tree to the schedulable process set.
  Step 12: it determines whether all the queues are empty. If yes, go to step 14. If no, go to step 13.
  Step 13: according to the process conflict adjustment strategy of the two-workshop vertical process tree constraints, it determines the processing workshop of the process and its actual start processing time and updates the schedulable process set; go to step 12.
  Step 14: it holds the substantial scheduling sequence results of all Root-Subtree processes.
  Step 15: the non-Root-Subtree processes in the stack space are sequentially popped out of the stack, and the non-Root-Subtree processes are added to the substantial scheduling sequence of step 14 to form a complete scheduling scheme for the product.
  Step 16: the product process tree Gantt chart is output.

### 5.2. Algorithm Complexity Analysis

It assumes that the number of the complex product processes is *n*, the number of the equipment is *m*, the number of the Root-Subtrees is *N*, and the number of the non-Root-Subtree processes stored in the stack space is *r*. The core of the proposed algorithm is to group and sort all Root-Subtree processes according to the single-workshop equipment sequence. On this basis, the process conflict adjustment strategy of the two-workshop vertical process tree constraints based on the principle of early processing is used to determine the processing workshop of the process and its actual start processing time.

1. Complexity analysis of the process conflict adjustment strategy of the horizontal equipment constraints: in the process of forming the Root-Subtree set, the worst case is that the process tree has only one leaf node, and the complexity of the tree set is *O*(*n*). According to algorithm ① and algorithm ②, the complexity of traversing each Root-Subtree to obtain the vertical and horizontal prescheduling completion time is *N* × *O*((*n* − *r*/*N*)^2^). The prescheduling scheme is selected according to the analysis results of the vertical and horizontal characteristics of the Root-Subtree, and the complexity of setting the priority parameters of the Root-Subtree using the bubble method is *m* × *O*((*n* − *r*/*m*)^2^).
2. Complexity analysis of the process conflict adjustment strategy of the two-workshop vertical process tree constraints. According to the process conflict adjustment strategy of the horizontal equipment constraints, the scheduling order of the Root-Subtree processes is determined and loaded into the corresponding queues in turn. The complexity of adding the schedulable processes to a schedulable process set is *O*(*n*^2^). In the worst case, the complexity of judging whether the first process of the queue is schedulable is *m* × *O*(*n*). When the first process of the queue is schedulable, it determines the processing workshop and the actual start processing time according to the different conditions of the processes, and the complexity of the first process of the queue being dequeued is *m* × *O*(*n*^2^). The complexity of the non-Root-Subtree processes being sequentially popped out of the stack and added to the scheduling sequence is *O*(*n*).

The two main strategies involved in the proposed algorithm are serial relations, and their complexity is the sum of the complexity of each strategy. The time complexity of the proposed algorithm is a quadratic polynomial *O*(*n*^2^).

## 6. Example Analysis and Algorithm  Comparison

### 6.1. Example Analysis

The proposed algorithm is a theoretical analysis process and does not depend on the product process tree structure. In order to better illustrate the execution process of the algorithm, the algorithm is used to conduct a scheduling test on a product instance to verify the universality of the algorithm in the distributed two-workshop integrated scheduling problem. It assumes that product H consists of 26 processes and needs to be processed collaboratively in workshop W1 (main workshop) and workshop W2 (slave workshop) with the same equipment resources. Each node contains three kinds of data information: process name, processing equipment and processing time, and the process migration time of *T*_*pm*_=1. The schematic diagram of the product process tree H and its split is shown in Figure 6. After the process tree is split, the formed Root-Subtree set is {*rt*_1_, *rt*_2_, *rt*_3_, *rt*_4_}.

After the Root-Subtree set is formed, it uses algorithm ① and algorithm ② to traverse each Root-Subtree, respectively, to obtain *T*_*Z*_^*rt*_*k*_^ and *T*_*H*_^*rt*_*k*_^. According to the comparison result of the prescheduling completion time, the prescheduling scheme is selected, and the priority of the Root-Subtree is set. The analysis process of the vertical and horizontal characteristics of the Root-Subtree set of the product H and the priority parameters of the Root-Subtree is shown in Table 2.

The Root-Subtree Priority Strategy determines the priority parameters of the Root-Subtree. At the same time, the specific information of the prescheduling start processing time of the Root-Subtree process grouped by a single-workshop equipment sequence is described as follows: M1: {A2:0, B1:15, C3:4, D4:5, D5:0}, M2: {A7:0, A4:4, B4:4, B3:8, C1:9, D1:12}, M3: {A3:12, B5:3, B6:0, C4:0, D2:8}, M4: {A6:0, A5:4, A1:17, B7:0, B2:7, C5:0, C2:6, D6:0, D3:4}. It uses the same equipment Root-Subtree process sorting strategy to establish the queues (Queue_1_, Queue_2_, Queue_3_, Queue_4_) combines the Root-Subtree priority strategy to determine the scheduling order of the Root-Subtree processes on the corresponding processing equipment, and loads them into the corresponding queues from front to back according to this order, the same equipment Root-Subtree processes of the product H are loaded into the corresponding queue, as shown in Figure 7.

After the operation of loading all the Root-Subtree processes into the corresponding queues is completed, the processing workshop of the process and its actual start processing time are determined according to the process conflict adjustment strategy of the two-workshop vertical process tree constraints. It generates the substantial scheduling sequence of the Root-Subtree processes, the specific analysis process to determine the processing workshop of all Root-Subtree processes, and their actual start processing time is shown in Table 3.

Finally, the non-Root-Subtree process in the stack space is taken out and added to the substantial scheduling sequence of the Root-Subtree processes to form the final scheduling scheme of product H so that it completes the product production scheduling task. The proposed algorithm is used to schedule product H, and the output Gantt chart is shown in Figure 8.

The following uses ISA-EPSP, ISA-TWOT, ISA-TPNR, and ISA-AEMA to schedule product H in Figure 6, respectively, and the superiority of ISA-CPRP is analyzed by comparing the sequence of process scheduling. When it uses ISA-EPSP and ISA-TPNR to schedule the products, it replaces the number of the process migrations with the process migration time, which can better reflect the consistency of the algorithms comparison results. The scheduling Gantt chart of ISA-EPSP, ISA-TWOT, ISA-TPNR, and ISA-AEMA is shown in Figures 9–12.

Figures 8–12 show that the total processing time of product H scheduled by ISA-CPRP is 26, and the total processing time of product H scheduled by ISA-EPSP, ISA-TWOT, ISA-TPNR, and ISA-AEMA is 27, 27, 29, and 27. By comparing the scheduling results of the five algorithms, ISA-CPRP fully exploits the vertical and horizontal characteristics of the process-associated positions in the process tree and improves the scheduling compactness of the process, and the production target can be better optimized. The main reason is that ISA-EPSP, ISA-TWOT, and ISA-TPNR all use a unified vertical or horizontal strategy to analyze and schedule processes as a whole and focus too much on load balancing and local optimization. It leads to the solidification of the processing workshop selection and scheduling order of the process, and it causes unnecessary process migration and idle time periods in some processes, which delays the actual start processing time of the process and affects the overall scheduling result of the product. For example, ISA-EPSP groups the schedulable processes into batches and uses the process balance strategy to determine the processing workshop. It focuses much on the process balance strategy and cannot consider the impact of the parent node on the process migration.  Figure 9 shows that the algorithm allocates process A3 to workshop W1 for the balance of the total processing time of the equipment, and the process migration makes the compactness between process A3 and process A5 worse. ISA-TWOT uses the long-path method to determine the process scheduling order and uses the two-workshop timing scheduling strategy to determine the processing start time of the process and the processing workshop to generate the optimal process scheduling plan, and it focuses much on the execution order of the local process sequence.  Figure 10 shows that the algorithm makes process C1 scheduled as soon as possible. It causes process C1 to be assigned to workshop W2, and the process migration makes the compactness between process C1 and the root node worse. ISA-TPNR uses the key equipment balance strategy and the long-path strategy to determine the processing workshop of the key equipment process and its scheduling sequence. It focuses much on the balanced treatment of the key equipment process and does not consider the impact of the key equipment process on the noncritical equipment process.  Figure 11 shows that the algorithm uses the key equipment balancing strategy to assign processes C5 and D6 to the same workshop and uses the long-path strategy to determine that process C5 is scheduled to be prioritized over D6, which causes the immediately following processes of process D6 in the Root-Subtree *rt*_4_ to be processed later so that it affects the overall scheduling result. ISA-AEMA searches all possible combinations according to certain constraints, which leads to slow solution efficiency, and it may evolve to the wrong area, which is easy to fall into local optimum and makes the searchability of the solution smaller.

### 6.2. Algorithm Comparison

In order to verify the performance of ISA-CPRP in the two-workshop collaborative, integrated scheduling problem and its adaptability to products with different structures, this paper randomly obtains 50 product instances with different structures that meet the integrated scheduling tree constraints. It requires that each product instance can be split into two to six Root-Subtrees.  Figure 13 depicts the comparison of ISA-EPSP, ISA-TWOT, ISA-TPNR, ISA-AEMA, and ISA-CPRP, scheduling 50 product instances, Figure 14 depicts the comparison of the average processing time to schedule 50 product instances using the above five algorithms. The figures show that the scheduling results of ISA-CPRP are better than the scheduling results of the other four algorithms. The experimental data results show that the more complex the product structure and the more Root-Subtrees, the better the scheduling effect of ISA-CPRP. The above description further confirms that it is necessary to excavate the internal structure of the product process tree in the two-workshop collaborative, integrated scheduling problem. It verifies the effectiveness and superiority of the proposed algorithm for solving the product instances with different structures.

## 7. Conclusion

In the integrated scheduling field, a two-workshop collaborative, integrated scheduling algorithm considering the prescheduling of the Root-Subtree processes is proposed for the first time and compared with the four existing two-workshop collaborative, integrated scheduling algorithms. The following conclusions are obtained:

1. The proposed algorithm uses the decomposition granularity control principle to split the product process tree into several Root-Subtrees and analyzes the vertical and horizontal characteristics of the Root-Subtree process at the associated position of the process tree by prescheduling. It uses the same equipment Root-Subtree process sorting strategy to determine the Root-Subtree process scheduling order by grouping the single-workshop equipment sequence and enhances the compactness of process scheduling.
2. This paper abandons the two-workshop equilibrium treatment strategy and uses the process migration time instead of the number of the process migrations, which more intuitively reflects the impact of the process migration on the scheduling results.
3. This paper proposes the process conflict adjustment strategy of the two-workshop vertical process tree constraints to solve the vertical process tree constraint relationship. On the basis of the vertical and horizontal analysis, the processing workshop and the actual start processing time of the process are determined. The strategy narrows the search comparison for schedulable processes to improve solution efficiency and improves the substantial parallel processing capability of process scheduling.
4. Compared with the existing algorithms, the proposed algorithm has better advantages in solving the two-workshop collaborative, integrated scheduling problem and truly achieves vertical and horizontal mergers.

To sum up, the idea of the proposed algorithm is to mine the vertical and horizontal characteristics inside the process tree in order to provide a reasonable scheduling scheme for various forms of product instances and expand a new direction for in-depth research on distributed two-workshop integrated scheduling problems.

## Figures and Tables

**Figure 1:** The schematic diagram of the modular product structure.

**Figure 2:** Schematic diagram of splitting product process tree O.

**Figure 3:** (a) The vertical and horizontal comparison of the Root-Subtree *rt*_1_ prescheduling Gantt chart. (b) The vertical and horizontal comparison of the Root-Subtree *rt*_2_ prescheduling Gantt chart. (c) The vertical and horizontal comparison of the Root-Subtree *rt*_3_ prescheduling Gantt chart.

**Figure 4:** The process conflict adjustment strategy of the two-workshop vertical process tree constraints.

**Figure 5:** The flowchart of the proposed algorithm.

**Figure 6:** The schematic diagram of the product process tree H and its split.

**Figure 7:** The schematic diagram of loading the same equipment root-subtree processes of product H into the corresponding queue according to the scheduling order.

**Figure 8:** ISA-CPRP schedules product H and outputs the corresponding Gantt chart.

**Figure 9:** ISA-EPSP schedules product H and outputs the corresponding Gantt chart.

**Figure 10:** ISA-TWOT schedules product H and outputs the corresponding Gantt chart.

**Figure 11:** ISA-TPNR schedules product H and outputs the corresponding Gantt chart.

**Figure 12:** ISA-AEMA schedules product H and outputs the corresponding Gantt chart.

**Figure 13:** Comparison of the total processing time to schedule 50 product instances by ISA-EPSP, ISA-TWOT, ISA-TPNR, ISA-AEMA, and ISA-CPRP.

**Figure 14:** Comparison of the average processing time to schedule 50 product instances by ISA-EPSP, ISA-TWOT, ISA-TPNR, ISA-AEMA, and ISA-CPRP.

**Table 1:** The same equipment root-subtree process scheduling sequence of the product process tree O.

Equipment sequence	Process name	Prescheduling start processing time	The priority parameter of the root-subtree to which the process belongs	The same equipment process scheduling sequence
M1	O6	10	*Q*_*rt*_^2^	2
	O8	20	*Q*_*rt*_^3^	4
	O9	20	*Q*_*rt*_^1^	3
	O13	0	*Q*_*rt*_^1^	1

M2	O4	45	*Q*_*rt*_^3^	4
	O7	10	*Q*_*rt*_^2^	3
	O10	0	*Q*_*rt*_^2^	2
	O12	0	*Q*_*rt*_^1^	1

M3	O3	45	*Q*_*rt*_^2^	2
	O5	75	*Q*_*rt*_^1^	3
	O11	0	*Q*_*rt*_^3^	1

**Table 2:** The specific analysis process of the priority of the root-subtree set of the product process tree H.

Root-subtree name	Vertical prescheduling completion time	Horizontal prescheduling completion time	$\frac{T_{Z}^{rt_{k}}}{T_{H}^{rt_{k}}}$	Number of the root-subtree process	The selected prescheduling scheme	Root-subtree priority
*rt*_1_	23	20	>1	7	Horizontal	*Q*_*rt*_^1^
*rt*_2_	20	17	>1	7	Horizontal	*Q*_*rt*_^2^
*rt*_3_	13	13	=1	5	Vertical	*Q*_*rt*_^4^
*rt*_4_	14	17	<1	6	Vertical	*Q*_*rt*_^3^

**Table 3:** The proposed algorithm determines the processing workshop of all root-subtree processes and their actual start processing times.

Equipment name	Process name	The initial start processing time	The final completion time of the two-workshop equipment	The reference start time for the two-workshop equipment	The selected workshop/the actual start time
M1	A2	0	0/0	—	Workshop W1/0
	D5	0	4/0	—	Workshop W2/0
	C3	8	5/4	9/8	Workshop W2/8
	D4	8	4/5	8/9	Workshop W1/8
	B1	18	10/10	19/18	Workshop W2/18

M2	A7	0	0/0	—	Workshop W1/0
	A4	4	2/0	4/5	Workshop W1/4
	B4	4	2/0	5/4	Workshop W2/4
	B3	8	7/7	8/9	Workshop W1/8
	C1	15	15/7	16/15	Workshop W2/15
	D1	16	15/19	17/19	Workshop W1/17

M3	B6	0	0/0	—	Workshop W1/0
	C4	0	3/0	—	Workshop W2/0
	B5	0	3/4	—	Workshop W1/3
	D2	12	8/4	13/12	Workshop W2/12
	A3	16	8/16	16/17	Workshop W1/16

M4	A6	0	0/0	—	Workshop W1/0
	B7	0	4/0	—	Workshop W2/0
	D6	0	4/4	—	Workshop W1/4
	C5	0	8/4	—	Workshop W2/4
	A5	2	8/8	8/8	Workshop W1/8
	D3	0	16/8	—	Workshop W2/8
	C2	10	16/12	16/12	Workshop W2/12
	B2	7	16/15	16/15	Workshop W2/15
	A1	21	16/18	21/22	Workshop W1/21

## Data Availability

The data that support the findings of this study are available from the corresponding author upon reasonable request.
